The article "Correlation between the Quality of Talent Training and Regional Economic Development Based on Multivariate Statistical Analysis Model" was retracted in 2023. Reasons: signs of a paper mill; suspected computer-generated content; unreliable results or conclusions; concerns about the data.

# Correlation between the Quality of Talent Training and Regional Economic Development Based on Multivariate Statistical Analysis Model

**DOI:** 10.1155/2022/2206689

**Published:** 2022-10-11

**Authors:** Yana Yuan

**Affiliations:** School of Economics and Management, Hainan Normal University, Haikou 571158, China

## Abstract

Entering the era of knowledge economy, the economic value of talent education is more and more emphasized, and it contributes more and more to the local economy and injects new vitality into local economic development. However, there are still some difficulties in the synergistic development of talent education and local economy, such as the low degree of integration of “industry, profession, and employment” and the lack of synergy between schools and enterprises, which affects the high-quality development of talent education and restricts the long-term development of regional economy. This paper incorporates machine learning algorithms to construct a multivariate statistics analysis model based on the correlation analysis model between talent training quality and regional economic development. Based on the multi-variate statistical analysis theory and method, the qualitative analysis and quantitative analysis are closely combined to scientifically pick up the main indicators affecting the comprehensive quality of talent cultivation and overcome the drawbacks of artificial subjective assignment of values. Through the judicious selection of evaluation indexes, a scientific and fair evaluation model is established, and the targets of talent cultivation are combined with regional economic development, in a comprehensive analysis, which provides a new means for the development of the regional economy.

## 1. Introduction

The normal function of the economy cannot be separated from talent, capital, land, technology, and other factors. In the beginning of economic development, there is often an adequate labor force [1], which ensures the direct contribution of labor as well as human capital to economic growth. This period can also be used to curb the process of diminishing returns to capital by shifting labor to increase the rate of resource allocation and effectively promote sustained economic growth. This is also known as the demographic bonus. The demographic dividend has played a considerable role in China's long periods of rapid economic growth after the reform and opening up [2]. It was only around the turn of the century that the demographic structure of our country began to show the characteristics of an aging society, labor is also becoming short, and the cost of labor for enterprises is raising, the influence of the traditional factors supporting economic growth is diminishing, and the bottleneck is coming [3]. Despite the demographic dividend generated by the quantity of the labor force disappearing, the quality of the working-age population, such as education, skills, and education experience, also offers a great potentiality for economic growth and is entering a new period of economic development in which the quality of the labor force is the main motivating factor.

The article "Correlation between the Quality of Talent Training and Regional Economic Development Based on Multivariate Statistical Analysis Model" was retracted in 2023. Reasons: signs of a paper mill; suspected computer-generated content; unreliable results or conclusions; concerns about the data.

For the nation's sustainable economic growth, scientific and technological progress, the number of labor force, and the improvement of the economic system are all essential and important factors [4]. A certain amount and quality of human capital is a more critical factor to bring the above influences to a reasonable level. Nowadays, the total labor surplus and temporary shortage of labor in China coexist, and there is a lack of labor with high quality and high skills. The overall level of human capital in China is still in an unreasonable state of uneven distribution and low quality; on the one side, China is facing an imbalance between labor supply and demand, and on the other side, it is exposed to the contrast between the low cultural quality and professional skills of the labor force and the backward level of human resource management, while generating the awkward situation of uneven distribution and large overall quantity of human capital in China [5]. And human capital shows a certain profit-seeking nature, human capital will flow to economically developed areas, which leads to the phenomenon of talent mobility. With low fertility levels, the country is no longer able to rely on the quantity of the workforce to drive economic development and must shift to a workforce quality-driven economy; thus, there is a demand to continuously improve the quality and skills of workers, increase total factor productivity, and transform China from a country with a large population to a country with strong human capital. Talent represents high-quality labor, the bearer of knowledge, and the creator of value; therefore, having talent is a source of inexhaustible capital power. The strength of a region's talent competitiveness has a great influence on its economic development, and human resources have become an important factor in economic development, which has received attention from various countries and regions. Our government attaches great importance to talent, and Secretary Xi Jinping frequently puts forward talent-related discourse, where he underlined how the competition of comprehensive national power is ultimately the competition of talents, and should improve the mechanism of talent development and establish a sound system of talent system, etc., and he notes the strong role of talent and the importance of maintaining its resources [6].

The article "Correlation between the Quality of Talent Training and Regional Economic Development Based on Multivariate Statistical Analysis Model" was retracted in 2023. Reasons: signs of a paper mill; suspected computer-generated content; unreliable results or conclusions; concerns about the data.

Education is an important way to form human capital, while vocational education is an essential part of education. Vocational education is principally about developing skilled human capital [7]. With the swift development of China's economy and society, the continuous optimization and upgrading of industrial structure has promoted the demand for highly skilled personnel. The recent increase in the number of technology-, knowledge-, and capital-intensive industries has made highly skilled personnel an increasingly important part of the workforce. The demand for talents at this stage mainly rests on the supply of vocational education talents, and vocational education plays a vital role in the long process of economic and social development. In the past few years, the State Council has proposed to accelerate the development of modern vocational education and gradually develop a vocational level education system with Chinese characteristics [8], such as adapting to the needs of industrial development, deepening the integration of industry and education, and coordinating vocational education with general education. The report of the 19th National Congress proposes to accelerate the development of modernization of vocational education, which can not only ease the pressure of employment but also provide more highly skilled personnel [9]. Studying the spatial effects of vocational education talent supply on economic growth based on human capital perspective and the imbalance in the geospatial distribution of human capital caused by many factors such as spatial heterogeneity and the level of economic development is taken into account to provide a theoretical basis for the formulation of policies related to the development of vocational education in China.

Recently, various regions in China are facing transformation and upgrading, and the target of competition is shifting from natural resources and capital to talents. Many first- and second-tier cities, such as Shenzhen, Xi'an, Nanjing, Changsha, and Tianjin, have introduced a number of talent attraction policies as a way to attract the majority of knowledge-based and skilled talent to come. Since 2016, the Shenzhen government has been dramatically relaxing the requirements for settling in the city and granting additional subsidies to college students who come to work in the city. Then, Changsha and Wuhan likewise adopted a policy of liberalizing their household registration and offering housing concessions. At the end of May 2017, the Xi'an Municipal Government issued 23 talent attraction policies, and it plans to invest heavily in attracting 1 million talents over a 5-year period.

The article "Correlation between the Quality of Talent Training and Regional Economic Development Based on Multivariate Statistical Analysis Model" was retracted in 2023. Reasons: signs of a paper mill; suspected computer-generated content; unreliable results or conclusions; concerns about the data.

Analyzing the major factors affecting the quality and attractiveness of talent training and correctly assessing the impact of the regional economy on the quality and attractiveness of talent training. National and international scholars have evaluated the attractiveness of talent in each region using various statistical methods. In this paper, by combing the existing literature, they study the correlation between the quality of talent training and regional economic development from various dimensions such as economic development environment, living service environment, and science and technology education environment. At this stage, talent has emerged as an important strategic resource for economic development, so we need to have a comprehensive understanding of the needs of regional economic development and the overall status of local development to attract talent. Second, this paper investigates both the number and structure of talents by combining the statistical methods of machine learning algorithms, qualitative, and quantitative and analyzes the role of its quantity on economic development, the degree of its structure, and industrial structure fit. Based on the above analysis, we are looking for a balance factor suitable for regional economic development and talent training quality.

## 2. Related Works

### 2.1. Interactive Development of Talent Quality and Regional Economy

Now, China's talent education shows a good development trend, deep development of human resources, to create a dividend of talent-driven regional economic development, which has made an important contribution to the local economy [10]. Serving regional economic development is one of the missions of local universities, and it is the path of common development for both local universities and regional society to establish a healthy interactive development relationship. In line with the transformation of the national economic structure, industrial structure, and economic development mode, it has become a common social concern how higher education institutions can play a role in participating in regional economic and social development [11]. Thus, many local universities focus their attention on improving the quality of talent cultivation to enhance the service capacity to the regional economy.

It is not merely the development trend of higher education but also the objective need of social development and the inherent requirement of national strategic development. The location and features of the university are in line with the development of the times and the real needs of social and economic construction and are also formed during the long-term development process of school operation. The rational positioning of the school and the deepening of its characteristics are the prerequisites for the realization of serving the regional economy, and the quality of talent training is the key to serve the regional economic development. In the time of the massification of higher education, the differentiation of social demand requires a clear hierarchy of talent cultivation [12, 13]. Local universities base on the needs of regional economic and social development, clarify the fundamental task of cultivating talents for regional social development, the specification of talent cultivation, and explore the innovation of talent cultivation system and new mode suitable for the positioning of local universities.

The article "Correlation between the Quality of Talent Training and Regional Economic Development Based on Multivariate Statistical Analysis Model" was retracted in 2023. Reasons: signs of a paper mill; suspected computer-generated content; unreliable results or conclusions; concerns about the data.

In line with the quick development of the country's economy, higher requirements have been put forward for talent training. To make the professional setting closer to the needs of economic and social development, while actively developing programs to restructure majors and build special majors, local schools should clearly understand that as a distinctive local teaching and research university, they should not merely foster applied innovative talents but also train top innovative talents, cultivate multi-disciplinary cross-composite talents such as engineering and management, and cultivate high-quality engineering and technology talents [14]; not only to fulfill the development needs of industries and enterprises but also to meet the regional economic and social development and the national economic demand for higher education, and even international needs; not only should the overall objectives of knowledge, ability, and quality be required but also provide different development directions according to students' individual development. Students will not only be able to perform general science and management work but also have the ability to innovate and will even become leaders in the industry. For this, a school should be based on its own advantages and specialties, should elaborate training programs, and provide diversified training of innovative talents [15].

Besides, to further complete the school-enterprise joint training mechanism, it needs to be oriented to the needs of society, with actual engineering as the background and engineering technology as the main line to focus on improving students' engineering awareness, engineering quality, and engineering practice ability. Make full use of the role of enterprises in the cultivation of engineering talents to promote students' engineering literacy, cultivate, and create a large number of high-quality engineering and technology talents with strong innovation ability and adapt to the needs of economic and social development focusing on cross-fertilization of disciplines and cultivate compound talents. The present development of society displays a highly diversified trend, which requires the school to produce talents with not only solid professional basic knowledge but also complex talents with broad foundation, interdisciplinary background, and national competitiveness. For this, the university's overall optimization of multidisciplinary innovative talent cultivation program and construct credit mutual recognition courses, set up a joint training course platform, and build a composite talent training program in accordance with the principle of emphasizing the foundation and cross-discipline.

The article "Correlation between the Quality of Talent Training and Regional Economic Development Based on Multivariate Statistical Analysis Model" was retracted in 2023. Reasons: signs of a paper mill; suspected computer-generated content; unreliable results or conclusions; concerns about the data.

### 2.2. Multivariate Statistical Analysis Methods and Their Main Types

The methodology of principal component analysis is the application of mathematical dimensionality reduction methods, whose intention is to replace the old variables with new ones, which are independent of each other, and to allow the user to decide whether or not to perform the distribution statistics [16]. Therefore, principal component analysis is a mode of analysis in which a few uncorrelated variables are replaced by a majority of correlated variables. The key feature of principal component analysis is that it can avoid the influence of set parameters and actual errors to the final statistical analysis results, and the analytic method selects more variables in the process of statistics, which improves the accuracy of the base size of the variables. Also, there are fewer variables in the process of analysis, and fewer variables do not affect each other; a process like this can make the statistical analysis results more consistent with the actual situation [17, 18].

The factor analysis method is an analysis method developed on the basis of principal component analysis, and its main target of study is the degree of connection within the matrix, that is, taking the matrix with the original index data as the basis, studying the internal structure of this matrix, and then searching for independent new factors that have a dominant effect on this structure so as to locate those particular factors that can influence the variables. The purpose of factor analysis is not to find the main factors [19, 20] but to know what these factors stand for. But the principal component analysis method finds the initial loading matrix of the solution of the principal factor that does not satisfy the simple structure principle and the typical variables represented by each factor are not very prominent, thus leading to ambiguity in the meaning of the factors. Therefore, it is not easy to explain economically by factors. For this, it is possible to rotate the factors to obtain satisfactory results [21].

The article "Correlation between the Quality of Talent Training and Regional Economic Development Based on Multivariate Statistical Analysis Model" was retracted in 2023. Reasons: signs of a paper mill; suspected computer-generated content; unreliable results or conclusions; concerns about the data.

The basic interpretation of cluster analysis is to summarize variables with similar properties by counting the distribution of variables and summarizing them in the analysis process so as to achieve a statistical approach for the purpose of reducing systematic variables. Actually, the cluster analysis method is a way to find a statistic, that is, a statistic that can objectively reflect the degree of close association between variables and classify these variables on that basis [22]. The two commonly used clustering statistics are coefficient of distance and similarity coefficient. However, there are three kinds of cluster analysis methods: systematic clustering method, tuning method, and graph theory method.

Statistical analysis of multivariate data is a branch of mathematical statistics that has emerged with the rapid development of computers, and its statistical analysis applications have been developed with the help of computers' superior data processing power, making statistical analysis easier, and allowing for larger volumes of data to be processed. The great data era has arrived, and multivariate statistical analysis methods have been applied to various areas of economic development. Statistical analysis of multi-variable data is focused on the theoretical and methodological application of the principles of mathematical and statistical methods, which leads to the study of multivariable problems, and it can simplify the complex Gini indicators and give a clearer picture of the meaning behind the economic indicators, which is also the most important utility of multivariate statistical analysis. Multivariate statistical analysis methods allow for variation and model construction without compromising existing information, which makes complex data simple.

## 3. Methodology

Figure 1 gives the schematic framework of the talent training quality and economic correlation analysis model based on the machine learning algorithm constructed in this paper. The three major modules include data pre-processing, machine learning model building and training, and correlation analysis.

### 3.1. Data Pre-Processing

The quality of data determines the accuracy of data digging outcomes to a large extent. Thus, data pre-processing techniques play a pivotal role in the data mining process [23]. In fact, a wide range of raw data sources, with missing value anomalies, noisy data, and inconsistent data, and these data can heavily compromise the quality and execution efficiency of data mining results, and may even lead to biased experimental results. Therefore, pre-processing operations such as cleaning, integration, transformation, and statute should be performed on the data before data mining to provide a reliable and standard dataset for later data analysis and mining.

The article "Correlation between the Quality of Talent Training and Regional Economic Development Based on Multivariate Statistical Analysis Model" was retracted in 2023. Reasons: signs of a paper mill; suspected computer-generated content; unreliable results or conclusions; concerns about the data.

#### 3.1.1. Data Cleaning

Data cleansing is the elimination of inaccurate, incomplete, inconsistent, and outlier data from a vast amount of raw data. Data cleaning is the most basic and time-consuming task in data pre-processing [24]. Generally speaking, the treatment of missing values primarily includes no treatment (the missing value has no effect on the data analysis), deletion (considering the amount of data with missing values), and data interpolation (the missing data is reasonably filled in). The most used operation for missing data completion in practical applications, and the common missing value completions are manual fill, average fill, and special value fill. Inconsistencies and outliers generally occur because the original data are stored in multiple databases or because of inconsistent data naming rules, and eliminate data inconsistencies by naming and specifying data consistently, which is also a prerequisite for data integration. The processing of outliers is generally handled legally using a delete or mean correction operation.

#### 3.1.2. Data Integration

To make data mining results more accurate and effective, we can integrate and summarize data from different data sources by using data from multiple data sources [25]. Due to the differences in data storage methods and data types, attention should be paid to the naming and formatting of each data source during the integration process, and attribute redundancy issues and entity identification issues should be fully considered.

#### 3.1.3. Data Transformation

Data conversion is mainly the normalization of data to form a data format that conforms to data mining methods, and the normative processed data are a fundamental task in the data mining process. Different source data often have various magnitudes and values, and the large variation of data objects can affect the data mining results to a large extent. Therefore, normalizing the data and scaling the attribute data to the scale to distribute its values in a specific area to facilitate data analysis of data objects. Commonly used data transformation methods contain min–max normalization and zero-mean normalization [26].

Min–max normalization [27]: the given data attributes are transformed to map them in the interval [0, 1]. Min–max normalization keeps the original relationships of data attributes of data objects and removes the problem of large differences in data levels and data ranges of data objects, as shown in equation (1).

(1) $$\begin{array}{c} v\_\text{data}=\frac{v-\min}{\max-\min}, \end{array}$$

where *v*_data indicates the data value of the data object after the min–max normalization process. *v* indicates the initial value of the data object; max and min denote the maximum and minimum values of the data object, respectively.

The article "Correlation between the Quality of Talent Training and Regional Economic Development Based on Multivariate Statistical Analysis Model" was retracted in 2023. Reasons: signs of a paper mill; suspected computer-generated content; unreliable results or conclusions; concerns about the data.

Zero-mean specification [28]: let the mean and variance of attribute *A* be $\bar{A}$and *σ*, respectively, change the value of attribute *A* to 0 mean and 1 deviation by data transformation, the calculation is shown in equation (2).

(2) $$\begin{array}{c} v\_\text{dat}{\text{a}}^{\prime }=\frac{v-\bar{A}}{\sigma }. \end{array}$$

Data discretization is the division of continuous data into small segments and puts these data in a discretized interval. Frequently used data discretization includes equal-width discretization, equal-frequency, and clustering discretization; the equal-width discretization is the division of data attribute values into intervals of the same width; frequency discretization is the placement of the same amount of data in each interval; and clumping discretization is performed by clustering the algorithm to obtain *k* clusters, and then labeling the classification values of each cluster.

#### 3.1.4. Data Statute

In practical applications, the data being analyzed are often characterized by a large volume of data and voluminous data sets comprise redundant data that is not relevant to data mining, which makes data analysis and mining time-consuming. Thus, the data size is reduced by relevant means before data analysis and mining, and the data attributes after data statute still maintains almost the integrity of the original data, and the volume of data is relatively small, so that the performance and efficiency of analysis mining on the statute dataset is greatly improved and produces almost identical analysis results. The data statute mainly includes the attribute statute and the record statute.

### 3.2. Machine Learning Algorithm-Based Talent Training Quality and Economic Relevance Analysis Model

#### 3.2.1. Text Mining Principle

From a technical point of view, text mining is a multifaceted research area involving meaning mining, information retrieval, keyword processing, multi-field screening, and many other elements. Text mining is an efficient mining tool that is both effective in extracting the deeper meanings and accurate in processing the effective parts of them. The text agglomerations in the application of text clustering technology mainly refer to the unified data objects that are judged and divided into multiple categories, which allows for a high degree of similarity in meaning between keywords while different data have opposite meanings. The categorization process is first of all a text feature extraction process. On this basis, text objects with similar keywords are divided into the same groups, and a clustering model is rebuilt according to the groups in turn; the analysis of the clusters is implemented using software description methods based on all the algorithms describing the clusters. The above process is shown in Figure 2.

The article "Correlation between the Quality of Talent Training and Regional Economic Development Based on Multivariate Statistical Analysis Model" was retracted in 2023. Reasons: signs of a paper mill; suspected computer-generated content; unreliable results or conclusions; concerns about the data.

#### 3.2.2. Text Classification Representation

Based on the principle of text mining technology, a support vector machine (SVM) is selected as the text clustering model construction method. The SVM model expresses the similarity degree of words in terms of spatial similarity. Using the vector calculation method of space to classify texts, the degree of similarity between texts can be calculated using spatial vectors. Calculating the cosine distance is a classical method for analyzing text similarity measures. In the SVM model [29], since the information in each text set must be converted into a variety of multidimensional data that the computer can process, the entire computer's text set is represented by a space vector function.

For a document set *D*_1_ = {(*T*_1_, *W*_1_), ..., (*T*_*n*_, *W*_*n*_)}, since *T*_*i*_ in a document collection is likely to seriously affect the text analysis due to its order and repetitiveness. To make it straightforward to understand, it is assumed that the document *T*_*k*_ ignores the order of documents and is not duplicated. At this point, the *n*-dimensional coordinates can be expressed as {*T*_1_, *T*_2_, ..., *T*_*n*_}, treating the weight {*W*_1_, *W*_2_, ..., *W*_*n*_} as a corresponding position and coordinate. The flow of SVM construction is shown in Figure 3.

Optimized data streams are commonly used in text mining for clustering analysis, and the necessary operation before performing stream clustering analysis on the text is to use a specific algorithm to perform similarity measures on the text. This paper uses the composite metric. The two correlation vectors in the model library can be represented as a document vector $\vec{d}=\left\{t_{1},t_{i},...,t_{n}\right\}$, *t*_*i*_ is the feature content of this model library, where *i* = 1, 2, 3, ..., *n*. The simulation of the similarity between vectors can be expressed as shown in equation (3).

(3) $$\begin{array}{c} d\left(d_{1},d_{2}\right)=\sqrt{{\left({\vec{d}}_{1}-{\vec{d}}_{2}\right)}^{2}}, \end{array}$$

where ${\vec{d}}_{1}$ and ${\vec{d}}_{2}$ represent the feature vectors of two documents in the model library, respectively, and *d*(*d*_1_, *d*_2_) denotes the Euclid distance. The Hermann distance between texts is calculated by equation (4).

(4) $$\begin{array}{c} d\left(d_{1},d_{2}\right)={\left({\left.{\vec{\;|\;d}}_{1}-{\vec{d}}_{2}\right|}^{k}\right)}^{1/k}, \end{array}$$

where *k* denotes the parameter in the Hermann distance, and when this parameter is 2, the Hermann distance and the Euclid distance can be obtained by one calculation. Next, we can use sine similarity to measure the similarity of two texts, the sinusoidal similarity between two vectors, that is, the vectors of correlation between talent training quality and regional economy, $\vec{v_{i}}$ and $\vec{v_{i+1}}$, is calculated as shown in equation (5).

(5) $$\begin{array}{c} \sin\left(\vec{v_{i}},\vec{v_{i+1}}\right)=\frac{\vec{v_{i}}\cdot \vec{v_{i+1}}}{\left\|\vec{v_{i}}\right\|\cdot \left\|\vec{v_{i+1}}\right\|}. \end{array}$$

The text similarity in the established data vector space model is measured by the sine similarity of two vectors ranging between 0 and 1. The association between two document vector similarity measures, that is, the quality of talent development and regional economy, can be expressed by equation (6).

(6) $$\begin{array}{c} jac\left(v_{1}-v_{2}\right)=\frac{x\cap y}{x\cup y}, \end{array}$$

where *x*∩*y* is the set of two documents with the same features, and *x* ∪ *y* is the set of all the contents of the two documents.

The article "Correlation between the Quality of Talent Training and Regional Economic Development Based on Multivariate Statistical Analysis Model" was retracted in 2023. Reasons: signs of a paper mill; suspected computer-generated content; unreliable results or conclusions; concerns about the data.

## 4. Experiment

### 4.1. Experimental Environment and Evaluation Index

The experimental runtime environment uses Intel(R) Core(TM) i7-8750H CPU@ 2.20GHz, the graphics card is NAIDIA GTX 1080Ti 16G RAM, python 3.7, and utilizes the pytorch deep learning framework. The optimizer uses Adam; the initial learning rate is 5 × 10^−4^, the weight decay factor is 0.0005, and the batch size is 32. The model training loss curve is shown in Figure 4. In Figure 4, when the number of model iterations epoch is 12, the loss curves of both the training and test sets tend to be smooth, indicating that the model has converged.

In this paper, considering the sparsity of the data, 60% of the data are selected as training data and 40% as testing data. The SVM model is treated as a base classifier, and the robustness and generalization capabilities of the model are evaluated using various predictors.

To investigate the effectiveness of this paper's model in analyzing, the association between talent development quality and regional economic development, accuracy, precision, recall, and *F*1 values is used. Each evaluation index is shown in Table 1, and the calculation is shown in equations (7)–(10).

(7) $$\begin{array}{c} \text{Accuracy}=\frac{tp+tn}{tp+fp+tn+fn}, \end{array}$$

(8) $$\begin{array}{c} \text{Precision}=\frac{tp}{tp+fp}, \end{array}$$

(9) $$\begin{array}{c} \text{Recall}=\frac{tp}{tp+fn}, \end{array}$$

(10) $$\begin{array}{c} f1=\frac{2pr}{p+r}. \end{array}$$

The article "Correlation between the Quality of Talent Training and Regional Economic Development Based on Multivariate Statistical Analysis Model" was retracted in 2023. Reasons: signs of a paper mill; suspected computer-generated content; unreliable results or conclusions; concerns about the data.

### 4.2. Association Mining Visualization

Taking into account that calculating the dissimilarity based on the same set of features between two vectors yields a rather general result. Thus, it is necessary to optimize the data stream clustering algorithm. The optimization data streaming clustering algorithm refer to the optimization of the input data to output the data that satisfy the conditions, and the visualization of the clustering division is shown in Figure 5. The sequential steps of initial clustering points, initial division, modification of clustering points, and re-division are indicated in the order of top to bottom and left to right. We can see that the weight-balanced mean centroid of each clustered object is calculated to derive the maximum distance between each clustered object and the centroid of and compare them with the corresponding clustered objects according to the minimum distance, and recalculate all the clustering center objects that have changed according to the optimized data. The process of the above two steps is cyclic at a time until the individual clustering centers no longer have any changes when performing the calculation. This yields a cluster of *k* individuals that satisfy the minimum variance accuracy criterion.

### 4.3. Analysis of Results

To authenticate the proposed correlation model based on the machine learner statistical model to evaluate and analyze the impact of talent training quality on regional economic development, a single random forest (RF) [30], a GBDT [31], and an Xgboost [32] were constructed in the same experimental setting, respectively. The first modeling is based on a number of factors related to talent development that affect regional economic development. And using historical data for training, we evaluate the prediction ability of the model by predicting the indicators of the regional economy and comparing them with the actual indicators. Comparing the model evaluation metrics accuracy, precision, recall, and *F*1, the comparison results are shown in Figure 6.

We can see that the prediction model proposed in this paper has a great improvement in all four metrics compared with the single random forest, GBDT, and Xgboost models, and the prediction accuracy is higher. It can also be seen that the classification effect of individual models for regional economic forecasting differs significantly from the real data, and even though the improved version or optimized model improves the final prediction to some extent, the core of the real decision of the model accuracy is the selection of multivariate statistical data features and the fusion of models. The main reason why multivariate statistical models are better than individual models is that multivariate statistical models integrate multiple classification models and they can adequately consider each algorithm to observe data from different data spaces and structures, and give full play to the advantages of different algorithms. From a model optimal perspective, individual model training runs the risk of falling into local minima, which may give rise to poor model generalization performance, the power fusion of multiple base learners can effectively reduce the probability of falling into local minima.

The article "Correlation between the Quality of Talent Training and Regional Economic Development Based on Multivariate Statistical Analysis Model" was retracted in 2023. Reasons: signs of a paper mill; suspected computer-generated content; unreliable results or conclusions; concerns about the data.

Figure 7 gives the time overhead of the model in this paper and all the comparison models, and we can see that the overall advantage of our model is obvious with better real-time performance, both in the training and testing phases. Especially, the training time overhead of the model in this paper is 11.2 s and the testing time overhead is 6.1 s. The time overhead of training falls by 3 s compared to the best-performing GBDT model among all comparison models.

### 4.4. Ablation Studies

To further verify the effect of different settings of the distance metric function on the overall performance of the model, we use the Euclid distance, edit distance (Ed), and cosine similarity (Cos) measures for clustering samples for clustering simulation, respectively, and the initial parameters of the algorithm remain the same, and the impact curves of different distance metric functions on the prediction performance are shown in Figure 8. We can see from that the obvious advantage of using Euclid over Cos and Ed. The dominant cause is the simplicity of the Euclid computation, where the distance metric is implemented for clustering and similarity features only by calculating the length of the line segment between two points. And cosine similarity does not consider the magnitude of the vectors but only their direction. Moreover, the structure is relatively complex and the time overhead is high for high-dimensional data. The two-editor distance, Ed, is usually used in the calculation of character similarity and needs to be normalized before calculation.

To check the effectiveness of various features for the overall performance, the combination of different features is, respectively, predicted, and the results are shown in Figure 9.

Here, in all, we considered the characteristics of education (A), degree of industrial development (B), culture (C), attraction policy (D), talent policy (E), economic environment (F), and government service concept and level of government (G). We can see from Figure 9 that the prediction model accuracy tends to increase as the number of features increases and the prediction accuracy is relatively high, especially when characteristics related to educational policies and cultural climate are taken into account.

The article "Correlation between the Quality of Talent Training and Regional Economic Development Based on Multivariate Statistical Analysis Model" was retracted in 2023. Reasons: signs of a paper mill; suspected computer-generated content; unreliable results or conclusions; concerns about the data.

## 5. Conclusion

Serving regional economic development is one of the missions of local universities. It is the only way for local universities and regional society to create a benign interactive development relationship for their common development. This paper establishes a multivariate statistical analysis model of the correlation between talent training quality and regional economic development with the assistance of machine learning algorithms, and it also introduces how universities base on regional economic development and incorporate the upgrading of the ability to serve regional economic development with talent training mode, which explores an excellent path of innovation in strengthening the service of regional economy and improving the quality of talent training in terms of diversified talent training mode innovation, strengthening practical teaching, and the combination of industry-university-research.

## Figures and Tables

**Figure 1:** Machine learning algorithm-based talent development quality and economic relevance analysis model.

**Figure 2:** Clustering analysis flow.

**Figure 3:** Structure of SVM model.

**Figure 4:** Model training curves.

**Figure 5:** Clustering visualization.

**Figure 6:** Comparison of prediction effects between different models.

**Figure 7:** Comparison of training and testing time overhead of different models.

**Figure 8:** Effect of different metrics on overall performance.

**Figure 9:** Effect curves of varying features on prediction performance.

**Table 1:** Confusion matrix.

	Actual	
Predicted	Positive	Negative
Positive	*Tp*	*Fp*
Negative	*Fn*	*Tn*

## Data Availability

The datasets used during the current study are available from the corresponding author upon reasonable request.
